The article "Exploration of the Value of Combined UA, IL-6, and fPSA/tPSA in the Diagnosis of Prostate Cancer" was retracted in 2023. Reasons: signs of a paper mill; compromised peer review; unreliable results or conclusions.

# Exploration of the Value of Combined UA, IL-6, and fPSA/tPSA in the Diagnosis of Prostate Cancer

**DOI:** 10.1155/2022/8542376

**Published:** 2022-03-09

**Authors:** Qionghua Tang, Zhijiang Liang, Yingchun Zhou, Yihui Huang

**Affiliations:** Department of Clinical Laboratory, The First Affiliated Hospital of Guangzhou University of Chinese Medicine, Guangzhou, Guangdong 510405, China

## Abstract

**Objective:**

To investigate the differences in uric acid (UA), interleukin-6 (IL-6), and free prostatic-specific antigen (fPSA)/total prostatic-specific antigen (tPSA) (F/T) between patients with and without prostate cancer (PCa) in order to discover the value of the three indicators in improving PCa diagnostic accuracy.

**Methods:**

Patients with pathologically diagnosed PCa (PCa group, *n* = 25), patients with other benign prostate diseases (benign group, *n* = 25), and men who underwent normal physical examination (control group, *n* = 25) at the First Affiliated Hospital of Guangzhou University of Chinese Medicine between October 2020 and January 2021 were included. The serum UA, IL-6, and F/T levels of participants in the three groups were measured, and the measured data were statistically analyzed.

**Results:**

There were statistically significant differences in IL-6 and F/T among the three groups (all *P* < 0.05), but there were no statistically significant differences in UA (*P* > 0.05). The area under the receiver operating characteristic (ROC) curve (AUC) for the three indicators was, respectively, as follows: PCa group-benign group 0.5416, 0.6776, and 0.6832; PCa group-control group 0.5432, 0.9536, and 0.9887; and benign group-control group 0.5000, 0.8784, and 0.9456. Logistic regression analysis indicated that IL-6 and F/T were independent predictors of PCa, with AUCs of 0.6776 and 0.6832, respectively, and a combined accuracy of 72.0%.

**Conclusion:**

These results suggest that IL-6 and F/T have a good detection effect for PCa screening. Compared with the detection of F/T alone, the combined detection of IL-6 and F/T can improve the diagnosis rate of PCa to a certain extent, providing effective guidance for the clinical diagnosis and treatment of patients. The value of UA needs to be further studied, and its feasibility in the diagnosis of PCa needs to be further explored.

## 1. Introduction

Prostate cancer (PCa) is the most common urinary system malignancy in elderly men [1]. Its development may be the result of the combination of personal factors, such as age, genetics, family history, obesity, and metabolic syndrome, and environmental factors, such as diet, lifestyle, and infection. In Western countries, PCa is the third leading cause of cancer death in elderly male patients, second only to lung cancer and bronchia cancer [2]. In China, with the continuous aging of the population and changes in dietary habits, the number of obese individuals and diabetic individuals has increased, and the base of the susceptible population has increased, resulting in a significant increase in the incidence of PCa in recent years [3, 4]. PCa patients often lack specific clinical manifestations in the early stage, and PCa is not easy to distinguish from benign lesions such as benign prostatic hyperplasia (BPH) and prostatitis. In addition, most patients initially respond to androgen deprivation but eventually develop hormone-refractory PCa, leading to late clinical treatment failure and death [5]. In the early stage, the 5-year survival rate for patients with PCa confined to the capsule can exceed 90% after active and effective treatment, and the 5-year survival rate is only 30% or lower when metastasis occurs [6]. Therefore, an early, accurate diagnosis and rational treatment are very important for PCa patients.

The article "Exploration of the Value of Combined UA, IL-6, and fPSA/tPSA in the Diagnosis of Prostate Cancer" was retracted in 2023. Reasons: signs of a paper mill; compromised peer review; unreliable results or conclusions.

To date, the most widely used serum marker for the diagnosis of PCa in clinical practice is prostate-specific antigen (PSA), which has a strong predictive value for PCa [7]. The widespread popularity of PSA testing, economic growth, and improvements in medical systems has also led to an increased detection rate of PCa. However, due to a high false-positive rate [8, 9], the guidelines published by the United States Preventive Services Task Force no longer use PSA as a routine screening method for younger males [10]. Additionally, during the detection process, PSA levels are very susceptible to the influence of multiple factors, and the obtained values are not specific enough to accurately distinguish between PCa and other diseases, such as BPH [11]. A study indicated that the ability of PSA alone to discriminate and detect gray zone results was limited, while free prostatic-specific antigen (fPSA) to total prostatic-specific antigen (tPSA), i.e., F/T ratio, had a significant advantage [12, 13].

UA is an end product of purine metabolism that is generated in the liver through a series of processes, such as the hydrolysis, deamination, and oxidation of purine compounds that are decomposed by the cells of the body [14]. The production and excretion of UA are balanced. However, with improvements in living standards, due to changes in factors such as dietary habits and the environment, excessive UA production or insufficient excretion results in an increase in UA. Studies have shown that UA, as a prooxidant, can affect the occurrence and development of PCa through oxidative damage and activation of oxidative stress [15]. In addition, Xue et al. showed that a high serum UA level is a risk factor for PCa and is highly correlated with the development of PCa [16]. It showed the close influence of high UA levels on prostate cell damage and carcinogenic progression.

The article "Exploration of the Value of Combined UA, IL-6, and fPSA/tPSA in the Diagnosis of Prostate Cancer" was retracted in 2023. Reasons: signs of a paper mill; compromised peer review; unreliable results or conclusions.

Mu et al. showed that the expression of IL-6 in PCa tissue was higher than that in BPH tissue, and that the expression of IL-6 was significantly higher in PCa tissues at clinical stages T3-T4 [17]. IL-6 is widely involved in the regulation of immune cells in the body, inflammation responses, and the occurrence and development of a variety of cancers [18]. IL-6 may become an effective biological indicator for PCa diagnosis and treatment and the assessment of patient prognosis.

UA, IL-6, and F/T levels are easy to assess and relatively stable. Although previous studies have reported a correlation between each indicator and the pathogenesis of PCa, there is a lack of data regarding the value of the three makers combined for the diagnosis of PCa in China. Therefore, this study will assess UA, IL-6, and F/T to explore their combined specificity and sensitivity for the diagnosis of PCa, to improve the PCa diagnosis rate.

## 2. Materials and Methods

### 2.1. General Information

A total of 50 patients who underwent prostate biopsy at the First Affiliated Hospital of Guangzhou University of Chinese Medicine between October 2020 and January 2021 were included. Among them, 25 patients were pathologically diagnosed with PCa (PCa group), and they were all clinically screened to exclude other systemic tumor diseases; 25 patients with other benign prostate diseases were pathologically diagnosed with non-PCa composed the benign group. In the same period, 25 males who underwent normal physical examinations were selected as the control group. Written informed consent was obtained from all the patients. The protocol was approved by the Medical Ethics Committee of The First Affiliated Hospital of Guangzhou University of Chinese Medicine.

### 2.2. Detection of Serum Tumor Markers and Combined Indicators

In the morning, 3 mL of fasting venous blood was collected from all patients into a vacuum blood collection tube containing coagulant. The blood was centrifuged at 4000 r/min for 5 min at room temperature, and the separated serum was separated. The levels of serum UA, IL-6, tPSA, and fPSA were determined by electrochemiluminescence (ECLIA) using a Roche Cobas E602 automatic ECLIA immunoassay analyzer. The protocol was performed in strict accordance with the instruction manual.

### 2.3. Statistical Analysis

Statistical analysis was performed using SPSS 23.0 software. Quantitative data that conformed to a normal distribution are expressed as the mean ± standard deviation (mean ± SD); differences between groups were assessed using the independent sample *t*-test. Stepwise binary logistic regression was used to perform multivariate analysis of significantly different variables to establish a logistic regression model for the joint prediction of PCa. The diagnostic efficacy of UA, IL-6, and F/T for PCa was compared by plotting receiver operating characteristic (ROC) curves, and differences were considered statistically significant when *P* < 0.05.

The article "Exploration of the Value of Combined UA, IL-6, and fPSA/tPSA in the Diagnosis of Prostate Cancer" was retracted in 2023. Reasons: signs of a paper mill; compromised peer review; unreliable results or conclusions.

## 3. Results

### 3.1. UA, IL-6, and F/T Levels in the Three Groups

The serum levels of UA, IL-6, and F/T in the PCa group were compared with those in the control group, and the IL-6 and F/T levels in the PCa group were significantly higher than those in the control group (*P* < 0.05). Additionally, the differences in IL-6 and F/T levels were statistically significant between the PCa group and the benign group, and the differences in IL-6 and F/T levels were statistically significant between the benign group and the control group (*P* < 0.05). In contrast, there were no statistically significant differences in UA levels among the three groups (*P* > 0.05) (Table 1).

(Assessed by the rank sum test; ^∗^*P* < 0.05 vs. control group, #*P* < 0.05 vs. benign group)

### 3.2. Risk Factors for PCa

Logistic analysis of IL-6 and F/T, which were statistically significant indicators, was performed to compare the PCa group and the benign group. The significance value for the logistic regression was less than 0.05, indicating that the model was statistically significant. The result indicated that IL-6 (OR = 1.073, 95% CI: 1.081-3.843) is a risk factor that differentiates PCa from benign prostate diseases, and F/T (OR = 0.092, 95% CI: 0.023-0.106) may be a protective factor (Table 2). In summary, in distinguishing the PCa group from the benign group, the combined detection of IL-6 and F/T improved the PCa diagnosis rate to a certain extent compared to F/T detection alone. The combined use of IL-6 and F/T is expected to provide effective guidance for the clinical diagnosis and treatment of patients and has certain diagnostic significance.

### 3.3. The Diagnostic Values of UA, IL-6, and F/T for PCa

ROC curves were performed to evaluate predicted risk values of UA, IL-6, and F/T for PCa diagnosis. The results showed when the state variable for the PCa group was 1 and that for the benign group was 0, AUC (UA) = 0.5416, AUC (IL − 6) = 0.6832, and AUC (fPSA/tPSA) = 0.6776 (Figure 1(a)). When the state variable for the PCa group was 1 and that for the control group was 0, AUC (UA) = 0.5432, AUC (IL − 6) = 0.9887, and AUC (fPSA/tPSA) = 0.9536 (Figure 1(b)). When the state variable for the benign group was 1 and that for the control group was 0, AUC (UA) = 0.5000, AUC (IL − 6) = 0.8784, and AUC (fPSA/tPSA) = 0.9456 (Figure 1(c)). The AUCs indicated that IL-6 and F/T had splendid primary screening abilities for PCa while the screening ability of UA was relatively limited. The IL-6 and F/T results were statistically significant, but the UA results were not statistically significant.

The article "Exploration of the Value of Combined UA, IL-6, and fPSA/tPSA in the Diagnosis of Prostate Cancer" was retracted in 2023. Reasons: signs of a paper mill; compromised peer review; unreliable results or conclusions.

A, ROC curves when the state variable for the PCa group was 1 and that for the benign group was 0; B, ROC curves when the state variable for the PCa group was 1 and that for the control group was 0; C, ROC curves when the state variable for the benign group was 1 and that for the control group was 0.

## 4. Discussion

In recent years, with improvements in the living standards of the Chinese people and the increase in the average life expectancy, the incidence and mortality of PCa have increased, and PCa is gradually becoming a major disease affecting the health and quality of life of Chinese men [19]. Serum PSA is currently an important indicator for the clinical screening of PCa. However, it only has organ specificity, not tumor specificity. The 2020 National Guidelines for the diagnosis and treatment of prostate cancer recommend puncture biopsy when PSA is >10 ng/mL, and that F/T values or other indications should be assessed when PSA ranges from 4-10 ng/mL (gray zone) [20].

There were studies which showed that the serum UA levels were independently positively correlated with the overall risk of prostate malignant tumors [16]. However, the specific mechanism by which blood UA levels are related to PCa development has not been fully elucidated. Therefore, although UA has the potential for use as an effective indicator in combination with PSA in the diagnosis of PCa, further studies are needed to investigate the effectiveness and rationality. In addition, some studies have shown that proinflammatory cytokines interleukin-6 and -8 contribute to prostate malignancy. IL-6 plays an important role in PCa proliferation, invasion, and metastasis [21]. Therefore, some clinical studies have used it as a target for the treatment of PCa. In this study, there was no statistically significant difference in UA levels among the three groups. The levels of IL-6 and F/T were higher in the PCa group than benign group and control group. Furthermore, multivariate logic analysis found that IL-6 is a risk factor for PCa, while F/T may be a protective factor. In addition, the ROC curve also suggests that IL-6 combined with F/T has a good effect on the diagnosis of PCa. Consequently, the combination of the two indicators, i.e., IL-6 and F/T, improved the sensitivity and specificity of PCa diagnoses when PSA values were in the gray zone.

The article "Exploration of the Value of Combined UA, IL-6, and fPSA/tPSA in the Diagnosis of Prostate Cancer" was retracted in 2023. Reasons: signs of a paper mill; compromised peer review; unreliable results or conclusions.

Some scholars believe that serum uric acid may be a risk factor for the occurrence and development of elderly prostate cancer patients [22]. However, the data obtained in this study do not support that conclusion, which may be due to the small number of included cases.

This study has certain limitations. (1) it is a retrospective analysis, which may increase the risk of selection bias. (2) The total number of patients enrolled was small, which may reduce the predictive value. The findings of this study should be verified in future studies.

## Figures and Tables

**Figure 1:** ROC curves for the UA, IL-6, and F/T.

**Table 1:** Comparison of the serum UA, IL-6, and F/T levels among the three groups.

Group	Number of participants	UA (*μ*mol/L)	IL-6 (ng/mL)	F/T
PCa group	25	378.84 ± 106.12	78.50 ± 63.47#	0.15 ± 0.07#
Benign group	25	385.16 ± 91.09	18.17 ± 15.67^∗^	0.18 ± 0.09^∗^
Control group	25	383.52 ± 57.48	10.31 ± 4.49	0.38 ± 0.11

**Table 2:** Multivariate logistic analysis results.

		*B*	Standard error	Wald	Degree of freedom	Significance	Exp (*B*)	95% CI of Exp (*B*)	
								Lower limit	Upper limit
Step 1^a^	IL-6	.026	.014	3.680	1	.048	1.073	1.081	3.843
	F/T	-9.968	4.738	4.427	1	.035	.092	.023	.106
	Constant	.620	.785	.625	1	.429	1.860		

^a^The variables entered in step 1: IL-6 and F/T.

## Data Availability

The data used to support the findings of this study are available from the corresponding author upon request.
